# Effect of Hydrocortisone on Intradialytic Hypotension: A Preliminary Investigational Study

**DOI:** 10.1155/2020/4987547

**Published:** 2020-05-05

**Authors:** Hussein H. Alhawari, Sameeha Alshelleh, Hussam H. Alhawari, Izzat Ahmad Alawwa, Saif Aldeen AlRyalat, Ahmad Mesmar, Khaled Ojjoh, Karem H. Alzoubi

**Affiliations:** ^1^Division of Nephrology, Department of Internal Medicine, School of Medicine, The University of Jordan, Jordan; ^2^Division of Endocrinology, Department of Internal Medicine, School of Medicine, The University of Jordan, Jordan; ^3^Department of Special Surgery, School of Medicine, The University of Jordan, Jordan; ^4^Department of Internal Medicine, School of Medicine, The University of Jordan, Jordan; ^5^Department of Clinical Pharmacy, Faculty of Pharmacy, Jordan University of Science and Technology, Jordan

## Abstract

**Introduction:**

Approximately 15 to 33% of all dialysis treatments are complicated by intradialytic hypotension (IDH). In this study, we tested the hypothesis that the intravenous administration of hydrocortisone prior to HD treatment could prevent IDH or at least decrease the drop in the blood pressure resulting from IDH.

**Methods:**

This study was approved by our local ethics committee/IRB (2017/87) and by the Jordan Food and Drug Administration (7/clinical/18). Additionally, it is registered on ClinicalTrials.gov (NCT03465007). In this preliminary investigational study, we screened all chronic hemodialysis patients at our clinic who were 18 years of age or older (*n* = 82) for IDH. There were 14 patients included in the interventional part of this study; patients were given IV hydrocortisone for 3 consecutive HD sessions, followed or preceded by 3 intervention-free sessions where they were given 5 ml of saline as a placebo.

**Results:**

The initial total sample size was 82 patients. The frequency of IDH at our clinic was 24.4%. Fourteen out of the 20 patients who were diagnosed with IDH agreed to enroll in the interventional part of our study. The mean age of the patients in the interventional part of our study was 53.5 years (±10.3). These patients included 5 (35.7%) men and 9 (64.3%) women. Upon comparing the number of hypotensive attacks with and without the hydrocortisone administration, we found a significant difference (*p* = 0.003) between the hydrocortisone and placebo treatments in which 12 (85.7%) patients had fewer IDH episodes with the hydrocortisone treatment than with placebo.

**Conclusion:**

This preliminary investigational study found that the administration of a stress dose of hydrocortisone prior to hemodialysis could be an effective measure for preventing or minimizing the risk of IDH episodes. Additional prospective studies on this subject are needed. Ruling out adrenal insufficiency in patients diagnosed with IDH is also crucial.

## 1. Introduction

Approximately 15 to 33% of all dialysis treatments are complicated by intradialytic hypotension (IDH), which is associated with possible serious consequences [1–4]. The Kidney Disease Outcomes Quality Initiative (KDOQI) and European Best Practice Guidelines (EBPG) define intradialytic hypotension as a decrease in systolic blood pressure by ≥20 mmHg or a decrease in mean arterial pressure by 10 mmHg, and this is associated with clinical events and the need for nursing interventions [5].

IDH is associated with increased all-cause mortality, cardiovascular morbidity and mortality, and other diseases including myocardial infarction, fluid overload/heart failure, and stroke [6].

Hemodialysis is considered a stressful event that requires a significant increase in ACTH and cortisol levels [7]. Serum cortisol starts to rise 3-4 hours after starting hemodialysis, it peaks at 6 hours, and it returns to the predialysis level 24 hours after dialysis treatment [8]. Hemodialysis could remove some of the already present serum cortisol and along with the supposed delay in adrenocortical response; this will put our HD patients at risk for adrenal crisis [8].

Based on above, we believe that hemodialysis patients will not have enough time to physiologically raise their cortisol level to cover the stress imposed by the HD treatment, and this could be one of the main contributing factors to the development of IDH. Therefore, in this study, we tested the hypothesis that the intravenous administration of 100 mg of hydrocortisone given 30 minutes prior to HD treatment could prevent IDH or at least decrease the drop in the blood pressure during HD treatment.

## 2. Methods

This study was approved by our local ethics committee/IRB (2017/87) and by the Jordan Food and Drug Administration (7/clinical/18). Additionally, it is registered on ClinicalTrials.gov (NCT03465007). All participants signed an informed consent form, first to participate in the screening for intradialytic hypotension, then to participate in the interventional part of the study. This study adheres to CONSORT 2010 guidelines [9].

### 2.1. Design

This preliminary investigational study was designed as a randomized, placebo-controlled, double-blind, crossover trial. All patients included in the interventional part of this study were given an IV of hydrocortisone for 3 consecutive sessions, followed by or preceded by 3 intervention-free sessions where we used saline via an IV as a placebo.

The patients were allocated to hydrocortisone or placebo as the first intervention randomly using Randomizer.org. Patients and the providing nurses were blinded to the intervention, and the doses were given by the nurses (either hydrocortisone or placebo) to the patient.

### 2.2. Assessments

This comparative study was conducted from March 2018 through September 2018 at Jordan University Hospital (JUH), a tertiary medical center in Amman, Jordan.

We screened all chronic hemodialysis patients who are 18 years of age or older (*n* = 82) at the HD clinic at our university hospital for intradialytic hypotension. We defined intradialytic hypotension based on the KDOQI and European Best Practice Guidelines definitions as a decrease in systolic blood pressure of ≥20 mmHg or a decrease in mean arterial pressure by 10 mmHg, providing that this is associated with clinical events and the need for nursing interventions [5].

The BP was measured 30 minutes before HD initiation, at the beginning of HD, and every thirty minutes thereafter. The occurrence of IDH was defined as any drop in BP during HD with respect to the lower BP reading between the BP thirty minutes prior to HD initiation and the BP at the beginning of HD. Two of the authors (A.M and K.O) supervised the whole process and were present during the whole time of hemodialysis sessions, and they were the ones who documented the clinical events associated with the drop in blood pressure and also checked the blood pressure with any associated symptoms in addition to the every thirty-minute blood pressure measurement. Symptoms included mainly dizziness and fatigue, and the clinical interventions included stopping the ultrafiltration, Trendelenburg positioning, and intravenous fluid boluses. The annotation of these episodes was blinded with respect to the intervention.

Twenty of the 82 patients were diagnosed with intradialytic hypotension based on the three HD sessions. Fourteen of the 20 patients agreed to enroll in our study, and 6 declined. We screened all 14 of the patients for adrenal insufficiency by first taking random early morning serum cortisol level measurements. Serum cortisol was determined by the ADVIA Centaur cortisol assay, a competitive immunoassay using direct chemiluminescent technology (Bayer Diagnostics, UCSF Clinical Labs-Chemistry, San Francisco, CA 94143, USA). The normal reference range for morning cortisol was determined to be 4.3–22.4 mcg/dl. Seven of the 14 patients had random morning cortisol level > 10 mcg/dl (>276 nmol/l) and were without clinical symptoms or signs of adrenal insufficiency other than intradialytic hypotension, so we did not further investigate these patients for adrenal insufficiency [10]. The other 7 patients had a random early morning cortisol level < 10 mcg/dl (<276 nmol/l), so we proceeded with performing the adrenocorticotropic hormone (ACTH) stimulation test to rule out adrenal insufficiency. Four of the 7 patients had a normal ACTH stimulation test result with the cortisol level rising to >18 mcg/dl (>497 nmol/l). The other 3 were diagnosed with adrenal insufficiency, given that no rise in cortisol > 18 mcg/dl (>497 nmol/l) was shown. One of these three patients was already taking chronic 5 mg/day oral prednisone, which explains his findings. All three were referred to the endocrinology clinic. ACTH level measurements and pituitary MRI were done, and the results were consistent with those of idiopathic central adrenal insufficiency. ACTH was determined by the Elecsys ACTH test system using a quantitative electrochemiluminescence immunoassay (ECLIA) (Roche Diagnostics, Indianapolis, IN, USA, 2010). The normal reference range for ACTH was determined to be 7.2–63.3 pg/ml. Two patients declined receiving oral steroid replacement therapy but agreed to proceed with our clinical trial, and the third patient was kept on his same dose of prednisone and agreed to proceed with our clinical trial.  Figure 1 details the flowchart of the patient inclusion protocol used in this study.

### 2.3. Intervention and Measurements

Each eligible participant was instructed to not change his medication schedule or his diet. We did not implement any other new intervention to help with the intradialytic hypotension during the study period.

After obtaining proper consents from patients, we proceeded with administering 100 mg of intravenous hydrocortisone or saline, which was given 30 minutes prior to the initiation of HD [11]. We measured the BP thirty minutes prior to starting HD, at the beginning of HD, and every thirty minutes thereafter. We used our own upper arm automated blood pressure device (Fresenius 4008S) for the blood pressure measurement, which is the normal routine at our HD clinic. Blood pressure measurements were performed by our regular HD nurses (blinded to the intervention). We obtained the age, weight, height, TSH level, and early morning serum cortisol level from each patient. We also performed an echocardiogram for patients who complained of any cardiac symptoms during their daily activities such as exertional shortness of breath.

### 2.4. Statistical Analysis

We used SPSS version 24.0 (Chicago, USA) to perform the statistical analysis in our study. We used the mean (±standard deviation) to describe continuous variables (e.g., age). We used the count (frequency) to describe other nominal variables (e.g., sex). *p* < 0.05 was assigned as the *α*. Data were assessed for normality using the Shapiro-Wilk test, histograms, and Q-Q plots.

We used the Wilcoxon signed-rank test to analyze the difference between the frequency of hypotensive attacks with and without the hydrocortisone administration, and we reported the results as the number of negative ranks (cases in which the frequency of hypotensive attacks with the intervention was less than the frequency of hypotensive attacks without the intervention), positive ranks (cases in which the frequency of hypotensive attacks with the intervention was more than the frequency of hypotensive attacks without the intervention), and ties (the frequency of hypotensive attacks with the intervention equals the frequency of hypotensive attacks without the intervention).

We used a paired sample *t*-test to analyze the mean blood pressure between each day with the intervention and the days without the intervention.

We used the Pearson test to analyze the correlation between the mean systolic blood pressure measurements and age, weight, and TSH and morning cortisol levels.

## 3. Results

The total sample size was 82 HD patients. The frequency of IDH in our clinic was 20/82 (24.4%). The frequency of adrenal insufficiency was 3/14 (21.4%) in the patients who were diagnosed with IDH and agreed to enroll in the interventional part of our study.

We included 14 patients with IDH in the second part (interventional) of our study. The statistical analysis of our study showed that the patients had a mean age of 53.5 years (±10.3 years). There were 5 (35.7%) men and 9 (64.3%) women included in this study. Eight (57.1%) of the included patients were known to have hypertension. Details of the patient sample included in the interventional part of the study are shown in Table 1.

Upon comparing the numbers of hypotensive attacks with and without the hydrocortisone administration, we found a significant difference (*p* = 0.003) as follows:

- Negative ranks (i.e., cases in which the frequency of hypotensive attacks with the intervention was less than the frequency of hypotensive attacks without the intervention): 12
- Positive ranks (i.e., cases in which the frequency of hypotensive attacks with the intervention was more than the frequency of hypotensive attacks without the intervention): 1
- Ties: 1

The frequencies of IDH episodes with and without the intervention for each patient and the characteristics of each patient are shown in Tables 2(a) and 2(b).

A comparison between mean SBP for the included sample at days 1, 2, and 3 with and without hydrocortisone showed no significant differences, as shown in Table 3.

We did not find any significant correlation between the mean blood pressure measurements and the age, weight, and TSH and morning cortisol levels of the patients.

Echocardiogram was done for nine out of the 14 patients who complained of any cardiac symptoms during their daily activities such as exertional shortness of breath. It showed ejection fraction ranging around 50-60% and normal to grade 1 diastolic dysfunction.

No side effects were reported during or after the administration of intravenous hydrocortisone.

## 4. Discussion

This randomized controlled, double-blind, crossover study showed that the intravenous administration of 100 mg of hydrocortisone given thirty minutes prior to starting treatment for HD could significantly decrease the number of IDH episodes in HD patients (*p* = 0.003).

The prevalence of IDH at our HD clinic was 24.3%, which is consistent with the prevalence of IDH in other studies [1–4].

IDH is associated with increased all-cause mortality, cardiovascular morbidity and mortality, and other diseases, including myocardial infarction, fluid overload and heart failure, and stroke [6].

Adrenal insufficiency is not uncommon in chronic HD patients, and IDH can be one of the nonspecific signs of adrenal insufficiency in chronic HD patients [12], so it is crucial to rule out adrenal insufficiency in these patients, in addition to the fact that these patients will also need a daily maintenance dose of glucocorticoids beside the glucocorticoid stress dosing prior to stressful events like hemodialysis [7, 13].

This IDH etiology could be attributed to different possible causes, such as an imbalance between ultrafiltration and intravascular volume refilling rate, abnormal adaptive responses to ultrafiltration, cardiovascular diseases, age, autonomic dysfunction, and diabetes [1, 14].

Common interventions to treat IDH could include reducing the ultrafiltration rate, UF modeling, cooling the dialysate, midodrine, intravenous normal saline, adjusting blood pressure medications, adjusting the dry weight, sodium modeling in the dialysate, and others [1, 15].

Midodrine could be an effective treatment for IDH, but it could be associated with higher long-term mortality [16]. A high dialysate sodium level could have some hemodynamic benefits in HD patients, but it will lead to sodium loading and more weight gain between HD treatments, which could eventually lead to more IDH episodes [17]. Cooling the dialysate could be an effective measure for lowering the frequency of IDH by promoting peripheral vasoconstriction, but there was a higher rate of feeling cold among all patients [18]. One case report was published when this study was running showing that fludrocortisone could be helpful for the treatment of IDH [19], but in this study, we studied hydrocortisone instead which has both glucocorticoid and mineralocorticoid activity.

A hydrocortisone dosage of 300-450 mg/day was given to critically ill patients requiring chronic renal replacement therapy, and this resulted in the normalization of serum sodium and potassium in 4 of the clinical cases [20].

The serum cortisol level starts to rise 3-4 hours after starting hemodialysis, it peaks at 6 hours, and it returns to the predialysis level 24 hours after dialysis treatment [8]. Hemodialysis could remove some of the already present serum cortisol and along with the supposed delay in adrenocortical response; this will put our HD patients at risk for adrenal crisis [8].

Long-term use of supraphysiologic doses of glucocorticoids, even if just intermittent, may have adverse effects on many major organ systems; however, the risk-benefit ratio of its use can be improved by careful monitoring and following of preventive strategies to minimize its potential side effects [21]. This would include providing appropriate immunizations prior to the institution of therapy, also assessment for the presence of any preexisting conditions whose control may be affected by glucocorticoid use such as diabetes mellitus and hypertension [22]. For example, in patients who develop steroid-induced hyperglycemia, adding insulin treatment or adjusting its dose is a common and effective treatment and the same applies to patients with hypertension by adjusting BP medications if needed.

Based on our literature review (PubMed and Google), there is no clinical trial that has studied the possible therapeutic effects of hydrocortisone in the prevention of IDH. We strongly believe that using intravenous hydrocortisone as mentioned above could be a breakthrough, as it is an inexpensive, safe, and available medication for the management of IDH.

Our study has some limitations. Our study has a small sample size, but despite this, we found statistically and clinically significant results. Longitudinal multicenter studies are needed to assess the morbidity and mortality benefits of this treatment for patients with IDH.

## 5. Conclusion

This preliminary investigational study showed that the administration of a stress dose of hydrocortisone prior to hemodialysis could be an effective measure for preventing or minimizing the risk of intradialytic hypotensive episodes. Additional prospective studies on this subject are needed to further evaluate this topic. Ruling out adrenal insufficiency in patients diagnosed with IDH is also crucial.

## Figures and Tables

**Figure 1:** The flowchart of the patient inclusion protocol used in this study.

**Table 1:** The included sample in the interventional part of the study.

	Mean	Standard deviation	Count	Column *N* (%)
Age (year)	53.5	10.3	14	
Sex				
Male			5	35.7%
Female			9	64.3%
DM				
No			7	50.0%
Yes			7	50.0%
HTN				
No			6	42.9%
Yes			8	57.1%
Weight (kilogram)	75.8	17.9		
Interdialytic fluid gain (liter)	3.8	1.7		
TSH (mIU/l)	2.6	2.0		
Morning cortisol (nmol/l)	277.0	153.5		

DM: diabetes mellitus; HTN: hypertension; TSH: thyroid-stimulating hormone.

**Table:** (a) Frequency of IDH episodes with and without the intervention for each patient

	Day 1	Day 2	Day 3	Day 1+HC	Day 2+HC	Day 3+HC
Patient 1	Y	Y	Y	N	N	N
Patient 2	Y	N	N	Y	Y	N
Patient 3	Y	Y	Y	N	N	N
Patient 4	Y	Y	N	N	N	N
Patient 5	Y	N	Y	N	Y	Y
Patient 6	Y	N	Y	N	N	N
Patient 7	Y	Y	Y	Y	N	Y
Patient 8	Y	Y	Y	N	Y	Y
Patient 9	Y	Y	Y	Y	N	Y
Patient 10	N	Y	N	N	N	N
Patient 11	Y	Y	N	N	N	N
Patient 12	N	Y	Y	N	N	N
Patient 13	Y	N	Y	N	N	N
Patient 14	Y	Y	N	N	N	N
Total	12	10	9	3	3	4

IDH: intradialytic hypotension; HC: hydrocortisone; Y: yes; N: no.

**Table:** (b) The characteristics of every patient listed in (a)

	Age (year)	Sex	DM	HTN	Weight (kilogram)	Interdialytic fluid gain (liter)	TSH (mIU/l)	Morning cortisol (nmol/l)	ACTH stimulation test	Adrenal insufficiency
Patient 1	37	M	N	N	53.5	4.2	1.8	311	Not indicated	N
Patient 2	51	F	Y	Y	95.5	3.5	2.8	45	Normal	N
Patient 3	60	F	Y	Y	95.0	4.0	4.2	419	Not indicated	N
Patient 4	70	F	Y	Y	85.0	3.5	4.3	202	Normal	N
Patient 5	45	F	N	N	65.0	3.3	0.8	319	Not indicated	N
Patient 6	63	F	Y	Y	73.0	3.3	1.9	555	Not indicated	N
Patient 7	51	F	N	Y	95.0	3.0	1.1	287	Not indicated	N
Patient 8	63	M	Y	Y	87.0	5.3	2.3	107	Normal	N
Patient 9	49	M	N	N	49.0	3.7	2.5	94	Abnormal	Y
Patient 10	45	F	N	N	49.0	1.0	1.5	199	Normal	N
Patient 11	38	F	N	N	60.0	4.5	8.6	417	Not indicated	N
Patient 12	65	F	Y	Y	93.0	3.5	2.2	493	Not indicated	N
Patient 13	52	M	Y	N	72.0	4.0	2.8	169	Abnormal	Y
Patient 14	61	M	N	Y	90.0	3.0	0.5	263	Abnormal	Y

DM: diabetes mellitus; HTN: hypertension; TSH: thyroid-stimulating hormone; M: male; F: female; Y: yes; N: no.

**Table 3:** A comparison between mean SBP for the included sample at days 1, 2, and 3 with and without hydrocortisone.

	Mean SBP (mmHg)	SD	Mean difference	SD	*p* value
Day 1					
Without HC	118	22.7	2.0	10.3	0.47
With HC	116	23.1			
Day 2					
Without HC	112	23.2	2.5	9.7	0.36
With HC	109	21.9			
Day 3					
Without HC	105	19.4	-6.3	12.2	0.09
With HC	111	22.9			

HC: hydrocortisone; SBP: systolic blood pressure.

## Data Availability

Data are available from the corresponding author upon request.

## Abbreviations

ACTH: Adrenocorticotropic hormone
IDH: Intradialytic hypotension
HD: Hemodialysis
KDOQI: Kidney Disease Outcomes Quality Initiative
BP: Blood Pressure
IV: Intravenous.

## References

[1] Reilly R. F. (2014). Attending rounds: a patient with intradialytic hypotension. *Clinical Journal of the American Society of Nephrology*.

[2] Yamamoto K., Kobayashi N., Kutsuna T. (2012). Excessive fall of blood pressure during maintenance hemodialysis in patients with chronic renal failure is induced by vascular malfunction and imbalance of autonomic nervous activity. *Therapeutic Apheresis and Dialysis*.

[3] Bégin V., Déziel C., Madore F. (2002). Biofeedback regulation of ultrafiltration and dialysate conductivity for the prevention of hypotension during hemodialysis. *ASAIO Journal*.

[4] Kuipers J., Oosterhuis J. K., Krijnen W. P. (2016). Prevalence of intradialytic hypotension, clinical symptoms and nursing interventions-a three-months, prospective study of 3818 haemodialysis sessions. *BMC Nephrology*.

[5] Kooman J., Basci A., Pizzarelli F. (2007). EBPG guideline on haemodynamic instability. *Nephrology Dialysis Transplantation*.

[6] Stefánsson B. V., Brunelli S. M., Cabrera C. (2014). Intradialytic hypotension and risk of cardiovascular disease. *Clinical Journal of the American Society of Nephrology*.

[7] Letizia C., Mazzaferro S., de Ciocchis A. (2010). Effects of haemodialysis session on plasma beta-endorphin, ACTH and cortisol in patients with end-stage renal disease. *Scandinavian Journal of Urology and Nephrology*.

[8] Tsuchida S., Sugawara H., Fukuchi S. (1970). Plasma cortisol level during hemodialysis with Kolff's artificial kidney. *The Tohoku Journal of Experimental Medicine*.

[9] Moher D., Hopewell S., Schulz K. F. (2010). CONSORT 2010 Explanation and Elaboration: updated guidelines for reporting parallel group randomised trials. *BMJ*.

[10] Hägg E., Asplund K., Lithner F. (1987). Value of basal plasma cortisol assays in the assessment of pituitary-adrenal insufficiency. *Clinical Endocrinology*.

[11] Derendorf H., Möllmann H., Barth J., Möllmann C., Tunn S., Krieg M. (1991). Pharmacokinetics and oral bioavailability of hydrocortisone. *Journal of Clinical Pharmacology*.

[12] Yoon J. W., Lee Y. K., Choi M. J., Ryu J. W., Koo J. R., Noh J. W. (2015). FP730PREVALENCE of adrenal insufficiency and method of ACTH stimulation in chronic hemodialysis patients. *Nephrology Dialysis Transplantation*.

[13] Yanase T., Tajima T., Katabami T. (2016). Diagnosis and treatment of adrenal insufficiency including adrenal crisis: a Japan Endocrine Society clinical practice guideline [opinion]. *Endocrine Journal*.

[14] Sułowicz W., Radziszewski A. (2007). Dialysis induced hypotension--a serious clinical problem in renal replacement therapy. *Medicinski Pregled*.

[15] Knoll G. A., Grabowski J. A., Dervin G. F., O'Rourke K. (2004). A randomized, controlled trial of albumin versus saline for the treatment of intradialytic hypotension. *Journal of the American Society of Nephrology*.

[16] Hammes M., Bakris G. L. (2018). Intradialytic hypotension: is midodrine the answer?. *American Journal of Nephrology*.

[17] Hussein W. F., Schiller B. (2017). Dialysate sodium and intradialytic hypotension. *Seminars in Dialysis*.

[18] Bullen A., Rifkin D., Trzebinska D. (2019). Individualized cool dialysate as an effective therapy for intradialytic hypotension and hemodialysis patients’ perception. *Therapeutic Apheresis and Dialysis*.

[19] Seo Y., Jeung S., Kang S. M., Yang W. S., Kim H., Kim S. B. (2018). Use of fludrocortisone for intradialytic hypotension. *Kidney Research and Clinical Practice*.

[20] De Souza S. P., Bezerra R., Andrade L., Seguro A. C. (2006). Combined therapy with dialysis and glucocorticoids in critically ill renal failure patients. *Nephrology Dialysis Transplantation*.

[21] Oray M., Abu Samra K., Ebrahimiadib N., Meese H., Foster C. S. (2016). Long-term side effects of glucocorticoids. *Expert Opinion on Drug Safety*.

[22] Hoes J. N., Jacobs J. W., Boers M. (2007). EULAR evidence-based recommendations on the management of systemic glucocorticoid therapy in rheumatic diseases. *Annals of the Rheumatic Diseases*.

